The article "Association between Rosacea and Cardiovascular Diseases and Related Risk Factors: A Systematic Review and Meta-Analysis" was retracted in 2024. Reasons: unreliable results or conclusions; concerns about the data; concerns about the peer review; concerns about the citations.

# Association between Rosacea and Cardiovascular Diseases and Related Risk Factors: A Systematic Review and Meta-Analysis

**DOI:** 10.1155/2020/7015249

**Published:** 2020-06-17

**Authors:** Yanmei Li, Linghong Guo, Dan Hao, Xiaoxue Li, Yujia Wang, Xian Jiang

**Affiliations:** Department of Dermatology, West China Hospital, Sichuan University, Chengdu 610041, China

## Abstract

**Background:**

Rosacea is a common inflammatory skin disorder. Several studies, but not all, have suggested a high prevalence of cardiovascular diseases (CVDs) in rosacea patients. This study is aimed at investigating the association between rosacea and CVDs and related risk factors.

**Methods:**

We performed a literature search through PubMed, Embase, and Web of Science databases, from their respective inception to December 21, 2019. Two reviewers independently screened the articles, extracted data, and performed analysis, following the PRISMA guidelines. Odds ratios (OR) or standardized mean differences (SMD) and 95% confidence intervals (CI) were calculated for outcomes. The included studies' quality was evaluated using the Newcastle Ottawa Scale (NOS).

**Results:**

The final meta-analysis included ten studies. The pooled analysis found no association between rosacea prevalence and the incidence of CVDs (OR 0.97; 95% CI 0.86-1.10). Rosacea was found to be significantly associated with several risk factors for CVDs (OR 1.17; 95% CI 1.05-1.31), including hypertension (OR 1.17; 95% CI 1.02-1.35), dyslipidemia (OR 1.34; 95% CI 1.00-1.79), and metabolic syndrome (OR 1.72; 95% CI 1.09-2.72). However, no association was found between rosacea and diabetes mellitus (OR 0.98; 95% CI 0.82-1.16). Among the biological parameters, a significant association was found between rosacea and total cholesterol (SMD = 0.40; 95% CI = −0.00, 0.81; *p* < 0.05), low-density lipoprotein cholesterol (SMD = 0.28; 95% CI = 0.01, 0.56; *p* < 0.05), and C-reactive protein (CRP) (SMD = 0.25; 95% CI = 0.10, 0.41; *p* < 0.05). We found no association between rosacea and high-density lipoprotein cholesterol (SMD = 0.00; 95% CI = −0.18, 0.18; *p* = 0.968) or triglycerides (SMD = 0.10; 95% CI = −0.04, 0.24; *p* = 0.171).

**Conclusions:**

Although no significant association was found between rosacea and CVDs, rosacea was found to be associated with several of related risk factors. Patients with rosacea should pay more attention to identifiable CVD risk factors, especially those related to inflammatory and metabolic disorders.

## 1. Introduction

Rosacea is a common, chronic inflammatory skin disease. It is characterized by flushing, persistent erythema, papules, pustules, telangiectasia, and phymatous changes affecting mainly the convexities of the face, with ocular involvement [1]. According to published data [2], the global adult prevalence of rosacea is about 5.46%. There is no significant sex difference in rosacea incidence. People between the ages of 45-60 are more susceptible. The complex pathomechanism of rosacea involves the interplay of genetic factors; dysregulation of the immune, vascular, and nervous systems; and environmental factors such as ultraviolet radiation, alcohol, and microorganisms [3]. Studies have shown that rosacea starts with an inappropriate innate immune response due to external stimuli. This response eventually leads to worsened inflammation and abnormal blood vessels. Upregulation of inflammation-related genes and infiltration of inflammatory cells are found in all rosacea subtypes, even in those with transient erythema [4]. The sebaceous glands, abundant in the centrofacial region, were also suggested to participate in the inflammatory process of rosacea, which is consistent with the clinical manifestation of centrofacial distribution [5].

The article "Association between Rosacea and Cardiovascular Diseases and Related Risk Factors: A Systematic Review and Meta-Analysis" was retracted in 2024. Reasons: unreliable results or conclusions; concerns about the data; concerns about the peer review; concerns about the citations.

Cardiovascular diseases (CVDs), especially coronary heart disease and stroke, are together the number one global death cause [6]. Risk assessment is a critical step in the current approach aimed at preventing CVDs. The main risk factors include diabetes mellitus (DM), hypertension, dyslipidemia, and metabolic syndrome (MS). The disrupted metabolism of lipids plays a crucial role in the development of CVDs. It affects not only the heart's circulation but also the peripheral and cerebral arteries. Accumulation of lipids or fibrous material in the intima of arteries causes atherosclerosis. Serum lipids are prone to form plaques on the affected intima. When such plaques detach, they might block important arteries, leading to ischemic events [6]. In some guidelines, biomarkers of inflammation, notably C-reactive protein (CRP), were added to traditional risk factors as potential predictors of CVDs, especially in patients at intermediate risk [7].

Accumulating evidence has shown that rosacea is a systemic disease. The association between rosacea and multiple comorbidities, including depression, migraines, gastrointestinal disorders, and autoimmune conditions, has been demonstrated [8]. Several investigators have suggested that rosacea might increase the prevalence of CVDs and related risk factors [9–14]. However, the evidence is limited and still controversial [15–18]. This discrepancy might be because the available evidence comes from studies with a small sample size and inadequate statistical power, using different study methods, and with publication bias. Mechanistically, vascular endothelial growth factor (VEGF)+405C/G polymorphism was reported to be significantly associated with rosacea and is also a risk factor for abnormal coronary microvasculature [19]. Moreover, the same pathways were previously shown to be active in rosacea and atherosclerosis, including increased cathelicidins, proinflammatory cytokines, and endoplasmic reticulum stress [18, 20, 21]. Considering that rosacea and CVDs are both chronic diseases involving an interplay between genetic and inflammatory elements, we thought it is necessary to perform a meta-analysis to explore the relationship between them and the CVD-associated risk factors.

The article "Association between Rosacea and Cardiovascular Diseases and Related Risk Factors: A Systematic Review and Meta-Analysis" was retracted in 2024. Reasons: unreliable results or conclusions; concerns about the data; concerns about the peer review; concerns about the citations.

## 2. Materials and Methods

This systematic review and meta-analysis was conducted in accordance with PRISMA guidelines.

### 2.1. Search Strategy

We searched PubMed, Embase, and Web of Science databases from their inception dates to December 21, 2019. Keywords for this search were as follows: (“rosacea”) and (“cardiovascular” or “metabolic syndrome” or “diabetes” or “hypertension” or “dyslipidemia” or “cholesterol” or “C-reactive protein”). In addition, we screened references in all retrieved articles to identify potentially eligible studies and evaluated them based on the inclusion and exclusion criteria. Only studies in English were included for assessment.

### 2.2. Inclusion and Exclusion Criteria

Studies were selected for the final analysis according to the following inclusion criteria: (i) studies evaluating the association between rosacea and CVDs and risk factors, (ii) case-control studies, and (iii) studies directly providing odds ratios (OR) for major CVDs and risk factors, or mean and standard deviation (SD) for biochemical factors, or giving original and sufficient data to calculate OR. The exclusion criteria were (i) studies of reviews, abstracts, case reports, or conference publications; (ii) studies of the repeated report of same research subjects or repeated publications; and (iii) studies not reporting relevant data or data not available.

### 2.3. Data Extraction

Two investigators (Y.L. and L.G.) independently reviewed literature, extracted data from each eligible study, and cross-checked, with disagreements resolved by consensus discussion with the third investigator (D.H.). The missing data were obtained by contacting the study author. The following clinical and demographic characteristics of included studies were extracted: (i) study characteristics including lead author, year of publication, and country; (ii) participant characteristics encompassing age, sample size, and diagnostic criteria for rosacea; and (iii) main outcomes including OR and 95% confidence interval for CVDs, including cardiovascular death (CD), CVD, major adverse cardiovascular events (MACE), peripheral atherosclerotic occlusive disease (PAOD), ischemic heart disease (IHD), myocardial infarction (MI), stroke, coronary artery disease (CAD) and heart failure (HF), and CVD risk factors (hypertension, DM, dyslipidemia, and MS). Mean and SD for biochemical indicators include high-density lipoprotein cholesterol (HDL-C), low-density lipoprotein cholesterol (LDL-C), total cholesterol (TC), triglycerides (TG), and CRP. In this study, the primary outcome was the association between rosacea and overall cardiovascular disease, while the secondary outcome was the relationship between rosacea and CVD-related risk diseases and the association of rosacea with biochemical indicators related to cardiovascular diseases.

The article "Association between Rosacea and Cardiovascular Diseases and Related Risk Factors: A Systematic Review and Meta-Analysis" was retracted in 2024. Reasons: unreliable results or conclusions; concerns about the data; concerns about the peer review; concerns about the citations.

### 2.4. Quality Assessment

The quality assessment was based on the Newcastle-Ottawa Quality Assessment Scale (NOS) for case-control studies [22]. Each article was judged based on eight items that consider the representativeness of study population, the comparability of cases and controls, and ascertainment of the exposure. High-quality articles can earn up to 9 points (the comparability question gets up to two points). The studies given more than 7 points were considered high quality. More than 5 points were included in the meta-analysis.

### 2.5. Statistical Analysis

Quantitative meta-analyses were performed using the software Stata 12.0 (Stata Corporation, College Station, TX, USA). OR and 95% CI were meta-analyzed to assess the strength of the association between rosacea and CVDs and susceptibility to major risk factors. For biochemical indicators, the mean and SD were pooled and analyzed for comparison. Heterogeneity was tested based on Cochrane's *Q* statistic (significant at *p* < 0.10) and the *I*^2^ test (significant at *I*^2^ > 50%). All meta-analyses were performed using a random effects model. To assess the impact of individual studies and to explain heterogeneity, we conducted a one-study removed sensitivity analysis. The risk of publication was assessed using Egger's test. *p* value of less than 0.05 was considered statistically significant.

## 3. Results

### 3.1. Search Results

A total of 641 studies were identified after the initial search. After removing duplicates, 316 potentially eligible records remained. Titles and abstracts of these articles were further screened, resulting in the selection of 26 potential publications. After reviewing the full text of these 26 studies, we selected for the final analysis, ten case-control studies that met the inclusion criteria, with a combined sample size of 97,456 patients (Figure 1).

### 3.2. Study Characteristics and Quality Assessment

The basic characteristics of the ten studies are shown in Table 1. The studies were published between 2014 and 2019. Four studies were conducted in European countries, two in the United States, and four in Asia. The mean age, which was reported in nine studies, ranged between 44 and 50.63 years. The sample size ranged between 46 and 53,927 patients. The quality assessment of the included studies is summarized in Table 2. Seven of the studies were considered as being of high quality, with a quality score of ≥7 points. Two studies were of moderate quality (7 > score ≥ 5 points).

The article "Association between Rosacea and Cardiovascular Diseases and Related Risk Factors: A Systematic Review and Meta-Analysis" was retracted in 2024. Reasons: unreliable results or conclusions; concerns about the data; concerns about the peer review; concerns about the citations.

### 3.3. Assessment of the Association between Rosacea and CVDs

Five studies, with 97,054 rosacea and 1,546,111 control cases, were included to assess the association between rosacea and the susceptibility for CVDs. The pooled analysis found no association between rosacea prevalence and the susceptibility for overall CVDs (OR 0.97; 95% CI 0.86-1.10) (Figure 2).

### 3.4. Meta-Analysis of Association between Rosacea and Diseases That Increase the Risk for CVDs

Seven studies, with 95,160 rosacea and 1,542,042 control cases, were included to assess the association between rosacea and the susceptibility to present with risk factors for CVDs. The pooled analysis found a significant association between rosacea and diseases that increase the risk for CVDs (OR 1.17; 95% CI 1.05-1.31). Our results show that for individual risk factors, the prevalence of hypertension (OR 1.17; 95% CI 1.02-1.35), dyslipidemia (OR 1.34; 95% CI 1.00-1.79), and MS (OR 1.72; 95% CI 1.09-2.72) is higher in rosacea patients than in the control group. However, there was no association between rosacea and DM (OR 0.98; 95% CI 0.82-1.16) (Figure 3).

### 3.5. Meta-Analysis of Association between Rosacea and Biological Indicators for CVD Risk

Four studies, with 337 rosacea cases and 457 controls, were included to assess the association between rosacea and biological indicators for CVD risk. Our results show that the levels of TC (SMD = 0.40; 95% CI = −0.00, 0.81; *p* < 0.05) and LDL-C (SMD = 0.28; 95% CI = 0.01, 0.56; *p* < 0.05) in rosacea patients were higher than those in the control group. However, no differences were found in HDL-C (SMD = 0.00; 95% CI = −0.18, 0.18; *p* = 0.968) and TG (SMD = 0.10; 95% CI = −0.04, 0.24; *p* = 0.171) between the two groups (Figure 4). The pooled results for CRP and hs-CRP showed that both were higher in rosacea patients (SMD = 0.25; 95% CI = 0.10, 0.41; *p* < 0.05), for CRP (MD = 0.37; 95% CI = 0.07, 0.67; *p* < 0.05) and hs-CRP (MD = 0.21; 95% CI = 0.03, 0.40; *p* < 0.05), respectively (Figure 5).

### 3.6. Sensitivity Analysis and Publication Bias

The result of sensitivity analysis by emitting a single study in each turn showed that there is no substantial change in the results, indicating good robustness of meta-analysis results (Figure 6). No significant publication bias was found (*p* = 0.200) (Figure 7).

The article "Association between Rosacea and Cardiovascular Diseases and Related Risk Factors: A Systematic Review and Meta-Analysis" was retracted in 2024. Reasons: unreliable results or conclusions; concerns about the data; concerns about the peer review; concerns about the citations.

## 4. Discussion

In this meta-analysis study, we found no significant association between rosacea prevalence and the incidence of CVDs (OR 0.97; 95% CI 0.86-1.10). Similarly, a large Danish cohort study of 5,993 rosacea patients found no association between rosacea and CVDs (HR 0.93; 95% CI 0.77-1.12) [23]. Several specific reasons apply to the interpretation of the current results. First, except that one study described a minimum follow-up time of 1 year [17], the remaining four studies [10, 12, 15, 16] did not provide the minimum follow-up time. Therefore, the follow-up period in the included studies may be too short to detect a rise in CVDs, especially for younger patients. Second, the severity levels of rosacea might affect CVD clinical outcomes. A study found that the CVD risk of moderate to severe rosacea was significantly higher than mild rosacea [11]. Furthermore, a meta-analysis study showed that the incidence of CVDs increased only in individuals with severe psoriasis [24]. This association might also be found in rosacea patients. However, few enrolled studies in our meta-analysis provided detailed information on the severity of rosacea in patients. Third, the lack of association might be related to drug intervention. Recently published studies have shown that tetracycline reduces the risk for vascular diseases in patients with rosacea. It is speculated that, as an inhibitor of metalloproteinases, the beneficial effect of tetracycline might be due to its anti-inflammatory properties [25]. Due to the above reasons and the limitations of available data, we believe that this result needs to be interpreted with caution.

We found significantly higher prevalence rates of hypertension, dyslipidemia, and MS among patients with rosacea. It might be related to the chronic inflammation in rosacea. MS is a group of classical cardiovascular risk factors, including central obesity, hypertension, dyslipidemia, and glucose intolerance/type 2 diabetes. Systemic inflammation is assumed to promote the development of MS [26]. Underlying inflammation and dysfunction of the arterial wall in rosacea might explain the development of hypertension [27]. From a different perspective, it was hypothesized that calcium channel blockers (CCBs) trigger rosacea. This assumption was based on the fact that CCB triggers the flushing reaction. However, a large observational case-control study found no association between either ACEIs or ARBs and the risk for rosacea [15]. The effect of antihypertensive drugs on rosacea needs further research. As for dyslipidemia, it is known that systemic inflammation can cause structural changes in lipoproteins, which negatively affect their ability to eliminate cholesterol [28]. Another cause might be associated with the decrease in paraoxonase-1 (PON1) level, an HDL-associated antioxidant enzyme. Lower serum PON1 activity has been demonstrated in both dyslipidemic patients and rosacea patients [29]. However, we did not find a significant association between DM and rosacea. A previous study suggested that patients with advanced DM have a reduced risk for rosacea because advanced DM is often accompanied by impaired vasodilation, whereas one of rosacea's key characteristics is vasodilation [30].

The article "Association between Rosacea and Cardiovascular Diseases and Related Risk Factors: A Systematic Review and Meta-Analysis" was retracted in 2024. Reasons: unreliable results or conclusions; concerns about the data; concerns about the peer review; concerns about the citations.

Furthermore, we found a significant association between rosacea and both CPR and hs-CRP. A test for hs-CRP is usually used to measure low-grade inflammation. Such inflammation is a chronic, subclinical, and systemic condition that contributes to the pathogenesis of many noncommunicable diseases like atherosclerosis. Both clinical and experimental studies have confirmed the important role of inflammation in the pathogenesis of rosacea [31]. A cross-sectional study found that hs-CRP was higher in patients with rosacea than in those with no skin disease (*p* = 0.001) [32]. All these indicate that, in analogy to psoriasis [33], the low-grade inflammation in rosacea might be systemic.

Recently, much attention has been paid to studying the role of lipid metabolism in rosacea patients. Transcriptome analysis of rosacea patients demonstrated significant upregulation of genes related to alcohol and lipid metabolism and sebaceous gland regulation [4]. We found a significant association between rosacea and the levels of TC and LDL-C, but no association with HDL-C or TG. In the bloodstream, cholesterol is transported as various lipoproteins, primarily LDLs. LDL-C is a generally acknowledged risk factor for atherosclerotic cardiovascular disease (ASCVD) [6]. One study found that a decrease in LDL-C was directly associated with a decrease in the risk for major vascular diseases. Such a proportional reduction was noted irrespective of the baseline LDL-C concentration [34]. Therefore, monitoring and controlling total cholesterol levels in patients with rosacea, especially the concentration of LDL-C, are likely to have cardiovascular benefits. HDL-C was once considered to be beneficial because of its ability to transport cholesterol to the liver for metabolism and its inverse relationship with the risk for developing CVDs. However, given that no benefit has been observed following clinical applications, the functional quality of HDL-C needs further study [35]. Taken together, we found that there may be a correlation between rosacea and abnormal lipid metabolism, although the cause-effect relationship is unclear. This prompts us to be alert to lipid metabolic disorder and related complications in patients with rosacea.

The article "Association between Rosacea and Cardiovascular Diseases and Related Risk Factors: A Systematic Review and Meta-Analysis" was retracted in 2024. Reasons: unreliable results or conclusions; concerns about the data; concerns about the peer review; concerns about the citations.

Our study has some limitations. First, heterogeneity and other confounding factors might have affected our findings. The results should, therefore, be interpreted with caution. Second, it would have been interesting to evaluate the association between different severity levels of rosacea or its different phenotypes and CVDs and related risk factors. This, however, was not possible due to the limited data. Third, the case-control design of the included studies makes it impossible to fully evaluate the cause-effect relationships.

## 5. Conclusion

The present meta-analysis indicates that although no significant association was found between rosacea and CVDs, rosacea was found to be associated with several CVD risk factors. Patients with rosacea need to pay more attention to identifiable risk factors, especially those related to inflammatory and metabolic disorders. A comprehensive understanding of the incidence of risk factors for CVDs in rosacea patients can inform future preventive practices and treatment recommendations. Therefore, it is necessary to conduct prospective studies to determine whether patients with rosacea should more closely monitor the known CVD risk factors.

## Figures and Tables

**Figure 1:** Flow diagram of the literature search and selection process.

**Figure 2:** Forest plot of the association between rosacea and overall cardiovascular diseases (CVDs) in case-control studies.

**Figure 3:** Forest plot of the association between rosacea and cardiovascular disease (CVD) risk factors in case-control studies.

**Figure 4:** Forest plot of the association between rosacea and lipid metabolism indicators in case-control studies.

**Figure 5:** Forest plot of the association between rosacea and C-reactive protein (CRP) in case-control studies.

**Figure 6:** Sensitivity analysis for primary outcome.

**Figure 7:** Publication bias based on Egger's test.

**Table 1:** Basic characteristics of included studies.

First author, year	Country	Age (mean ± SD)	Rosacea (no.)	Control (no.)	Match factors	Rosacea subtype	Rosacea diagnosis	CVDs and related risk diseases	Reference
Sinikumpu, 2019	Finland	46	146	278	Gender, BMI, and tobacco use	Erythematotelangiectatic, papulopustular, phymatous, and ocular rosacea	ICD-10	N/A	13
Marius, 2019	Romania	47.87 ± 15.11	46	39	Age and gender	Erythematotelangiectatic and papulopustular rosacea	National Rosacea Society criteria	MS, HBP	14
Son, 2018	Korea	47.21 ± 15.01	2,536	1,396,992	N/A	N/A	ICD-10	IS, PAOD, IHD, DLP, DM, HBP	12
Belli, 2017	Turkey	50.63 ± 8.45	85	90	Age, gender, and BMI	Erythematotelangiectatic and papulopustular rosacea	N/A	MS	18
Egeberg, 2016	Denmark	49.2 ± 14.5	4,948	23,823	Age, gender, and calendar time	N/A	ICD-10	CD, MACE, IS, MI, HS, DM, HBP	16
Marshall, 2016	USA	49.1 ± 9.0	2,090	4,263	Age and gender	N/A	ICD-9	CVD,DM,	17
Rainer, 2015	USA	50.6 ± 14.1	65	65	Age, gender, and race	Erythematotelangiectatic, papulopustular, phymatous, and ocular rosacea	National Rosacea Society criteria	MS, HBP	11
Hua, 2015	China, Taiwan	44	33,553	67,106	Age and gender	N/A	ICD-9	IS, PAOD, CAD, DLP, DM, HBP	10
Duman, 2014	Turkey	44.65 ± 12.9	60	50	Age and gender	Erythematotelangiectatic, papulopustular, phymatous, and ocular rosacea	National Rosacea Society criteria	N/A	9
Spoendlin, 2014	UK	N/A	53,927	53,927	Age, gender, general practice, and calendar time	N/A	N/A	IS/TIA, MI, IHD, HF, DLP, DM, HBP	15

BMI: body mass index; N/A: not applicable; CD: cardiovascular death; CVDs: cardiovascular diseases; MACE: major adverse cardiovascular events; IS: ischemic stroke; TIA: transient ischemic attack; PAOD: peripheral atherosclerotic occlusive disease; MI: myocardial infarction; IHD: ischemic heart disease; CAD: coronary artery disease; HS: hemorrhagic stroke; HF: heart failure; HBP: hypertension; DM: diabetes mellitus; DLP: dyslipidemia; MS: metabolic syndrome.

The article "Association between Rosacea and Cardiovascular Diseases and Related Risk Factors: A Systematic Review and Meta-Analysis" was retracted in 2024. Reasons: unreliable results or conclusions; concerns about the data; concerns about the peer review; concerns about the citations.

**Table 2:** Quality assessment of the included studies.

Study	Selection				Comparability	Exposure			Total score
	Adequate definition of the cases	Representativeness of the cases	Selection of controls	Definition of controls	Control of important factors	Ascertainment of exposure	Same method of ascertainment for cases and controls	Nonresponse rate	
Duman, 2014	∗	—	—	∗	∗	∗	∗	—	5
Belli, 2017	∗	∗	—	∗	∗∗	∗	∗	—	7
Sinikumpu, 2019	∗	∗	—	∗	∗∗	∗	∗	—	7
Rainer, 2015	∗	∗	∗	∗	∗∗	∗	∗	—	8
Spoendlin, 2014	∗	∗	∗	∗	∗∗	∗	∗	—	8
Egeberg, 2016	∗	∗	∗	∗	∗∗	∗	∗	—	8
Hua, 2015	∗	∗	∗	∗	∗∗	∗	∗	—	8
Marshall, 2016	∗	∗	∗	∗	∗∗	∗	∗	—	8
Son, 2018	∗	∗	—	∗	—	∗	∗	—	5
Marius, 2019	∗	∗	—	∗	∗	∗	∗	—	6

## Data Availability

All the underlying data in the article are available online.
